The article "Risk Factors and Treatments of Suprachoroidal Hemorrhage" was retracted in 2023. Reasons: suspected computer-generated content; unreliable results or conclusions; lack of ethics approval or compliance; missing or withdrawn patient consent.

# Risk Factors and Treatments of Suprachoroidal Hemorrhage

**DOI:** 10.1155/2022/6539917

**Published:** 2022-07-14

**Authors:** Huaiyan Jiang, Yang Gao, Wenzhong Fu, Hongxia Xu

**Affiliations:** The First People's Hospital of Yunnan Province (Kunhua Hospital Affiliated with Kunming University of Science and Technology), Kunming, China

## Abstract

Suprachoroidal hemorrhage (SCH) is a rare but serious sight-threatening complication of inner eye surgery. Despite continuous advances in treatment, visual prognosis remains poor. The disease has a more typical clinical presentation, the etiology and pathogenesis are not well defined, and intraoperative ocular and systemic factors may induce fulminant SCH. To investigate risk factors and treatments of SCH-associated intraocular surgeries, summarize diagnosis, characteristics, management, and prevention of SCH developed during and after intraocular surgeries. A retrospective study of SCH occurred in six cases of intraocular surgeries including cataract, glaucoma, pars plana vitrectomy (PPV), and silicone oil removal surgery. Assess baseline systemic and ocular characteristics of SCH eyes. Analyze the second surgery timing and technique, and visual outcomes were measured. SCH occurred in six patients including five eyes during surgeries and one eye after the surgery. Three eyes that underwent cataract surgery had hard nucleuses (nuclear sclerotic 4+). One eye was due to hypotony during the vitrectomy procedure. One eye developed SCH when silicone oil was extracted from the eyeball. One eye developed delayed SCH after glaucoma surgery. Incision closure and anterior chamber deepening were performed. B-scan ultrasonography was used to diagnose SCH, and determine the timing and location of sclerotomy for the second surgery. Vitrectomy and sclerotomy were performed in five eyes. The median follow-up time was six months. The final best-corrected visual acuity (BCVA) was 0.3 in one eye, one eye had light perception with retinal adherence, and four eyes had no light perception with retinal detachment. The results showed that risk factors including advanced age, hypertension, taking anticoagulants, antiplatelet drugs, and cardiovascular drugs were systemic risk factors, and hard nucleus (nuclear sclerosis 4 +) cataract, long-term uncontrolled ocular hypertension glaucoma, vitrectomy, silicone oil removal, high myopia, aphakia, previous intraocular surgery, intraocular pressure during surgery, and others were ocular risk factors. The most important risk factor is a sudden drop in intraocular pressure during or after surgery. The outcome of visual acuity depends on retinal status. Because of the poor prognosis, the prevention of SCH is of utmost importance during intraocular surgery.

## 1. Introduction

The etiology of suprachoroidal hemorrhage (SCH) can be varied, with choroidal neovascularization being an important cause, seen primarily in macular lesions of age-related macular degeneration and high myopia, often with hemorrhage close to the macular area causing sudden loss of central vision. In addition, central exudative chorioretinopathy, acute choroiditis, optic disc edema, traumatic choroidal rupture, idiopathic polypoid cholangiopathy, and systemic diseases, such as hypertension, arteriosclerosis, hepatopathy, and diabetes, may result in choroidal hemorrhage. In addition to the above situation, the choroid also has a serious massive fulminant bleeding, called choroidal fulminant hemorrhage [1].

SCH mostly comes from the supply artery of the choroid, namely, the posterior ciliary artery. Pathological studies have found necrosis and rupture of the posterior ciliary artery in the affected eyes. There are several risk factors as follows. (1) In the clinical and pathological reports of glaucoma, many cases have glaucoma. (2) Hypertension and arteriosclerosis are common in the elderly and have varying degrees of arteriosclerosis and hypertension, so it may be one of the important factors of this disease. However, it is also reported that congenital cataracts in infants and young people occur during surgery. (3) Other systemic and eye diseases such as diabetes, hemorrhagic quality, polycythemia, and vascular fragility, as well as eye diseases such as high myopia, central retinal vein occlusion, and choroidal angiosclerosis, exist. 4. The problems related to the surgical operation are cut too quickly during the internal eye operation, and the intraocular pressure suddenly drops to the atmospheric pressure level, which can lead to rupture and bleeding of the great choroidal vessels or posterior ciliary artery from the sclera into the superior choroidal cavity. Inappropriate extrusion of the eyeball during the operation, resulting in excessive loss of vitreous, has the possibility of increasing the occurrence of this disease [2, 3].

Suprachoroidal hemorrhage (SCH) is a rare but blinding complication of any intraocular surgical procedure, including cataract, glaucoma surgery, penetrating keratoplasty, scleral buckling, and vitrectomy. SCH is a serious complication arising during (burst SCH) and after (delayed SCH) surgery in various types of inner eye surgeries (incidence 0.03%-6.10%) and can also occur spontaneously (spontaneous SCH, rare). SCH is defined as the accumulation of blood within the potential space of the choroid and sclera, with the source of the blood being the long or short posterior ciliary artery. It happens during or after the intraocular surgery unprepared and suddenly. The surgeon must pay attention to risk factors to avoid SCH. If it happens, unfortunately, handling it in a timely and careful manner is necessary [4].

## 2. Materials and Methods

This is a retrospective report of six cases (six eyes) of intraocular surgery who suffered SCH from 2014 to 2020, and the second surgery was performed on five eyes. The clinical materials were reviewed. The risk factors associated with SCH and the time when SCH developed in the intraocular surgeries were measured. We managed SCH through the blood drainage combined with PPV surgery. The timing and the location of the sclerotomy in the second surgery depended on the B-ultrasonography examination. The outcome of the ocular status and the best-corrected visual acuity (BCVA) were analyzed in our study. The clinical workup for SCH mainly includes laboratory tests as well as other ancillary tests: (1) laboratory tests: carry out laboratory tests related to the primary disease such as diabetes mellitus and bleeding disorders, such as blood glucose, bleeding, and coagulation indicators, and (2) other auxiliary examination: choroidal hemorrhage with sudden onset and stable condition can be considered for ultrasonography after it is clear that the condition of retinopathy is caused by choroidal hemorrhage.

## 3. Results

This is a retrospective study of SCH that occurred in intraocular surgeries performed in the Kunhua Hospital affiliated with Kunming University of Science and Technology from 2014-2020. There are six patients (six eyes): three males and three females. Their ages range from 69 to 78, and the mean age is 73.3. The preoperative best-corrected visual acuity (BCVA) was two 20/70: two fingers counted and two light perceptions, respectively. It included three cataracts, one glaucoma, one cataract combined with macular epimembrane, and one silicone oil tamponade eye. Three patients had hypertension. One eye was high myopia, and two eyes were monophthalmia. The glaucoma eye and the silicone oil tamponade eye had to elevate intraocular pressure (IOP) accompanied by optic atrophy.

The time of SCH occurred during the surgery in five eyes and after the surgery in one eye. Three cataracts had hard nucleuses (nuclear sclerotic 4+). The posterior capsular rupture took place in all three cases so the surgeon had to change the method from phacoemulsification to extracapsular cataract extraction (ECCE). SCH developed after the hard nuclear segment was extracted from the enlarged incision. The fourth eye of glaucoma surgery related to SCH occurred on the first day after the operation of Ahmed's glaucoma valve implantation, with a shallow anterior chamber postoperatively. The fifth case of SCH developed in the macular epimembrane eye during the vitrectomy procedure, and sudden ocular hypotony happened during fluid-gas exchange. The sixth case of SCH took place during the surgery of the extraction of silicone oil. It was ten years since the first vitrectomy, and elevated uncontrolled IOP developed before the surgery.

When SCH happened, all patients felt an ocular pain, nervousness, and headache. Intraocular pressure increased suddenly, intraocular contents were prolapsed, vitreous hemorrhage appeared, and one or two swellings were seen from the choroid. Once SCH was considered, the first step was to suture the surgical incisions promptly; prolapsed vitreous or nonviable iris tissue may need to be surgically excised to help wound closure. The anterior chamber was deepened by injecting a viscoelastic agent after repositioning any expulsed intraocular contents.

After the first operation, every patient had high IOP with pain and poor VA (no light or light perception). We treated it with antiglaucoma medications and steroids to prevent inflammation and promote clot liquefaction. After the first operation, B-scan ultrasonography was used to show the sign of choroidal swelling and “kiss choroidal” to confirm the diagnosis of SCH and locate the position of the suprachoroidal blood. Every two days, B-scan ultrasonography was performed to determine the timing of the clot liquidation and the location of the blood cavity, as shown in Figures 1–3. We performed second drainage surgery during the clot liquefaction shown by B-scan ultrasonography in five eyes for about 10-14 days. The patient underwent silicone oil removal but did not receive the second surgery because the SCH was localized in one quadrant, and there was no blood in the vitreous cavity. In the second surgery, a 1-2 mm long draining sclerotomy in a radial direction was made which was 4-10 mm from the limbus. The position of sclerotomy depended on the B-scan ultrasonography in the quadrant that contained the largest collection of blood. IOP could be controlled by limbal infusion. Vitrectomy was performed during the draining procedure of the SCH. In all 5 cases, perfluorocarbon liquid (PFCL) was used to force blood extrusion from the suprachoroidal space out through the sclerotomy incision, helping to remove more liquefied blood. In four eyes, we choose silicone oil instilled to provide an internal tamponade to reduce rebleeding into the suprachoroidal space, and in one eye, we choose viscoelastic injection in the vitreous cavity to prevent the postoperative hypotony. After 6 months of follow-up, the best-corrected visual acuity was 0.3 in only one eye, one eye had light perception, and 3 eyes had no light perception, as shown in Table 1. Postoperative anatomic status of the eyes was noted by B-scan ultrasonography and we found that the VA of two of the cases was over light perception with retina flattened and that of the rest cases was no light perception with retinal detachment, as shown in Figures 4 and 5.

## 4. Discussion

There are six consecutive cases with SCH developed in the intraocular surgery in this retrospective study. It is shown that the risk factors include advanced age, hypertension, taking anticoagulation, antiplatelet agents, and cardiovascular drugs which are the systemic risk factors [5] and hard nucleus (nuclear sclerotic 4+) cataract, glaucoma with uncontrolled high IOP for a long duration, vitrectomy, silicone oil removal, high myopia, aphakia, previous intraocular surgery, hypotony in the surgery, and so on which are the ocular risk factors [6, 7]. The most significant risk factor is the IOP drop down suddenly in the surgery or after the surgery. When we are aware of the SCH occurrence, we should keep calm and suture closure of the incision combined with withdrawing the iris and deepening the anterior chamber to resist the active bleeding [8, 9]. B-scan ultrasonography is important for the diagnosis of the SCH. We could also use it to determine the timing of the secondary drainage surgery. Some authors classify the SCH into 4 grades by the B-scan ultrasonography [2–4]. The first grade could not undergo the drainage surgery, and the other higher grades should perform the second surgery [2–4].

The second surgery of the SCH is controversial [1, 2, 4]. The timing of the second surgery of drainage is when liquefaction forms in the clot under the choroidal space. We choose surgical drainage combined with vitrectomy [2–8]. The combined vitrectomy with radial sclerotomy is the second surgical procedure in SCH. It clears vitreous hemorrhage, and the left lens segments prevent retinal detachment and vitreous traction complications. Drainage sclerotomy is usually performed after anterior chamber infusion placement [1, 2]. We mostly choose to perform radial sclerotomy at the position of 4-10 mm from the limbus depending on the location of the B-scan ultrasonography [2, 8, 10]. The liquefied blood under the choroidal space was drained successfully from the scleral incisions and kept the incision sutureless [1, 2, 4].

In the PPV process, we used perfluorocarbon (PFCL) to instill into the vitreous cavity. It forced more liquefied blood to drain from the radial scleral incisions when it sank to the posterior pole of the eyeball and extrude all other fluids anteriorly (such as blood within the suprachoroidal space). Therefore, PFCL was used to flatten the retina and choroid as other authors have suggested [1, 2, 4, 11]. When the retina and the choroid of the posterior pole flattened, we choose to use silicone oil in 4 cases and viscoelastic in one case for tamponade. Silicone oil provides sufficient filling and plays an anti-inflammatory role, and it could also protect against PVR [1, 2, 11]. Keeping a normal IOP is another function of silicone oil in several studies [1, 2, 11, 12]. It is reported that persistent hypotony is present in most cases of SCH [13, 14]. Despite these cases, all 5 cases underwent secondary surgery to keep normal IOP in our study. We believe that silicone oil prevents persistent hypotonia in the postoperative time [2–9]. Some authors reported that the viscoelastic is approved for intraocular use in posterior segment surgery of the SCH [15].

Once SCH occurs, we should first use various methods to control the bleeding to achieve the purpose of preserving eyesight and eyeball. More attention should be paid to prevention. Generally, measures should be taken to close the wound in time. If the bleeding cannot be stopped, the sclera can be cut open at the 8~10 mm behind the limbus, and the suprachoroidal hemorrhage can often be saved [10, 11]. To prevent the occurrence of SCH, a comprehensive examination should be performed before the operation, including vascular fragility and blood coagulation function test, control of blood pressure and intraocular pressure, and the light operation to avoid excessive overflow of eye content. (1) Usually pay attention to rest, and do not use your eyes too much. (2) Keep good living habits, get enough sleep, and do not stay up late. Avoid operating the computer continuously for a long time, pay attention to the rest in the middle, and usually operate continuously for 1 hour and then rest for 5-10 minutes. You can look at the distance or do eye exercises during the rest. (3) Usually be careful not to glare directly into the eyes. In addition, prevent eye trauma. Actively treat the primary disease so as not to cause SCH. (4) Maintain a good working posture. Maintain the most appropriate posture so that the eyes look flat or slightly down at the screen, which relaxes the neck muscles and minimizes the area of the eyeball exposed to the air [12–15].

The risk factors of SCH in intraocular surgery are hard nuclear cataracts, glaucoma, and vitrectomized eyes. It is reported that the significant risk factor for the SCH is both hypotony and increased intraocular pressure [3, 10, 13, 14, 16]. In the hard nuclear cataract, we use phacoemulsification to thin the full-thick nuclear and then perform a horizontal chop to divide it into two pieces, then four pieces, and so on. We must try to avoid the hard thick nuclear rolled over in the capsule, because the hard thick nuclear segment rolling over in the capsule is easy to cause the posterior capsular rupture [5]. The management of the complication may lead to hypotony and SCH. In glaucoma surgery, it is important that we could use viscoelastic to fill the anterior chamber at the end of the surgery. The technique can avoid the IOP decreasing in the follow-up [7, 9, 14]. In the vitrectomy surgery, we could pay more attention to maintaining stable IOP throughout the surgery to prevent the SCH from happening [6–17]. The visual outcome of SCH depends on the presence of retinal detachment. Following up with the SCH fading away, we should study the retina status and function [10].

## 5. Conclusion

SCH of intraocular surgery is disastrous and a vision-threatening complication. It may occur during intraocular surgery or after the surgery. The poor outcome of the visual acuity is the consequence of the retinal detachment [11–18]. In the first operation, we should proceed cautiously, using appropriate techniques, to avoid the occurrence of SCH. Pay more attention to high-risk cases. Prompt recognition and proper management may limit the consequences of SCH and provide a reasonable visual outcome for many patients. B-scan ultrasonography is useful for the diagnosis of SCH and the judgment of the timing and location of reoperation. In most cases, surgical draining combined with PPV is necessary for the second operation.

It is well known that the outcome of visual acuity depends on the presence of retinal detachment. As far as this study is concerned, there are still many limitations because the number of data for these cases of this study is small, and we need to collect more cases to summarize the experience and thus prevent and treat SCH [2, 4, 10, 18].

## Figures and Tables

**Figure 1:** B-scan ultrasonography reveals massive suprachoroidal hemorrhage with kiss choroidal central and retinal apposition. The macula is spared.

**Figure 2:** B-scan ultrasonography reveals massive suprachoroidal hemorrhage with the hemispherical bulge.

**Figure 3:** B-scan ultrasonography reveals massive suprachoroidal hemorrhage; the blood enters the vitreous.

**Figure 4:** B-scan ultrasonography of the patient 6 weeks after drainage with radial sclerotomies. Note that the hemorrhage has been cleared from the suprachoroidal space, but the retina is detached.

**Figure 5:** B-scan ultrasonography of the patient 12 weeks after drainage with radial sclerotomies. Note that the suprachoroidal hemorrhage has been cleared from the suprachoroidal space, but the retina is detached. And the visual acuity is NLP.

**Table 1:** Patients' demographics and clinical features.

Patient	Age (year)	Sex	VA IOP (pre-op)	Diagnosis	Time	Second drainage	VA (post-op)	Filling material (post-op)	Retinal detachment
1	70	Male	HM/20 cm 21 mmHg	Cataract Hypertension	During	Undergone	NLP	Silicone oil	Yes
2	70	Female	LP 22 mmHg	Cataract High myopia	During	Undergone	LP	Silicone oil	No
3	70	Female	HM/30 cm 19 mmHg	Cataract	During	Undergone	NLP	Silicone oil	Yes
4	70	Male	0.25 18 mmHg	Cataract Macular membrane	During	Undergone	0.3	Viscoelastic	No
5	70	Male	0.3 48 mmHg	Glaucoma	After	Undergone	NLP	Silicone oil	Yes
6	60	Female	LP 46 mmHg	Silicone oil tamponade Secondary glaucoma	During	No	NLP	Saline	No

## Data Availability

The simulation experiment data used to support the findings of this study are available from the corresponding author upon request.
